The article "Brent Crude Oil Price Forecast Utilizing Deep Neural Network Architectures" was published in 2022. Journal: Comput Intell Neurosci.

# Brent Crude Oil Price Forecast Utilizing Deep Neural Network Architectures

**DOI:** 10.1155/2022/6140796

**Published:** 2022-05-05

**Authors:** Amir Daneshvar, Maryam Ebrahimi, Fariba Salahi, Maryam Rahmaty, Mahdi Homayounfar

**Affiliations:** ^1^Department of Information Technology Management, Electronic Branch, Islamic Azad University, Tehran, Iran; ^2^Department of Industrial Management, Electronic Branch, Islamic Azad University, Tehran, Iran; ^3^Department of Management, Chalous Branch, Islamic Azad University, Chalous, Iran; ^4^Department of Industrial Management, Rasht Branch, Islamic Azad University, Rasht, Iran

## Abstract

Brent crude oil is considered as one of the most important sources of crude oil pricing in the worldwide market, and it is used to set the price of two-thirds of the traded crude oil supplies in the world. To predict the price of Brent crude oil, LSTM and Bi-LSTM methods are applied, which are the architecture of the recursive neural network. Initially, the database creates the appropriate data for the period January 2015 to March 2021 from Brent crude oil price signals and daily data from a financial market, and then, the modeling process is performed via the use of MATLAB software. Also, about 90% of the data are for training and the remaining for validation and comparison. Using LSTM and Bi-LSTM neural networks, the network architecture has been worked on, and by adding the number of layers and changing the solvers (SGDM, RMSProp, and Adam), the errors of different models are compared with each other. Nonlinear techniques of artificial neural networks and deep learning were used for modeling. Then, the network architecture was worked on and the model error rate was evaluated by comparing different layers and solvents such as SGDM, RMSProp, and Adam. The superiority of SGDM solvent over others was shown, and finally, it can be mentioned as the superior method of modeling of price forecasting in Brent crude oil field. The results show that the model with two layers of LSTM and SGDM solver has less error and better accuracy.

## 1. Introduction

Oil is a very important energy source whose international price fluctuations affect all aspects of the economy. The exchange rate is one of the important channels that shows how the international oil price shock is reflected in the real economy and financial markets. Understanding the characteristics and trends of oil price fluctuations provides the basis for a deep understanding of system mechanisms and the gradual trend in related research. Given the very complex characteristics of oil prices, it is very difficult to make accurate forecasts [1]. Men naturally seek to decipher the phenomena around the past in order to be able to predict the behavior of such phenomena and react to possible future events [2, 3]. It is more obvious in economic terms. The main feature of markets today is change, and the world is witnessing new developments and innovations in human societies. The highly dynamic nature and constant changes in the capital market have led researchers and economists to think about the best ways to predict the future and make the right decisions [4, 5].

In addition, models are used for analysis, better understanding, forecasting, systems development, etc., and basically in many financial issues such as investment and risk, the upper limit of the final quality of solving a problem is determined. Since price signals have a complex physical structure and it is very difficult to extract the laws and factors governing these signals, especially in the global scale, its effective parameters are not precisely defined and calculated, so analytical modeling are not appropriate. The purpose of this study was to present a model (or models) in a financial field by which the future price of Brent crude oil can be predicted with appropriate accuracy (minimum error). This issue will be modeled through the deep learning method. Using artificial intelligence and machine learning tools, a nonlinear model (or models) of artificial neural networks will be presented for price prediction. The most popular and widely used type of recursive neural network (RNN) is long short-term memory (LSTM). LSTM networks are able to solve the two main problems that exist in RNN, namely the disappearance slope and the explosion slope. The key to solving these problems is the internal structure used in LSTM. Here, LSTM and bidirectional long-short term memory (Bi-LSTM) are applied for the phase of modeling. Meta-heuristic methods such as colonial competition algorithm (CCA) or methods such as cross-validation will be used to optimize network parameters. The research hypotheses are as follows:

- The price signal contains information in its content
- The future price of time-series data is highly dependent on its past price
- The future price of time-series data depends on external factors related to it
- The performance of an expert system depends on the quality of its training

Additionally, the authors are looking for the way how financial market time-series data can be predicted through deep learning method.

In the following, in Section 2, the research background is examined.  Section 3 describes the research method. In Section 4, the results are numbered and analyzed, and finally in Section 5, conclusions are made.

## 2. Literature Review

Behradmehr [6] used wavelet transform and neural networks for New York crude oil and Gulf of Mexico crude oil over a period of low volatility to present a model with a more accurate prediction of New York crude oil prices and Gulf of Mexico crude oil than other models. In this hybrid model, the wavelet transform was used to reduce the noise level of the data and then the oil price was predicted by artificial neural networks with smoothed data. The results of this study indicated that the elimination of noise improves the performance of oil price forecasting. In another study conducted by Pourkazemi and Asadi [7], oil prices were predicted and compared using artificial neural networks and the ARIMA econometric linear model, which showed less error in neural networks. In this study, by adding the OECD countries' reserves as an input, the forecasting error is reduced.

Investigating the price gap of Brent crude oil and diesel fuel using econometric methods, neural networks and wavelet transform were performed by Zolfaghari et al. [8]. The purpose of this study was to investigate the factors affecting the price gap and test the principle of symmetry between Brent crude oil prices and diesel fuel prices. Based on the results of linear and nonlinear models in this study, the principle of symmetry is accepted in short-term fluctuations in crude oil prices. This is not the case with long-term fluctuations. Brent oil price forecast in 2013 was done by an innovative and combined method that was meta-analyzed registered at Urmia University [9]. The results of this study showed that the accuracy of the meta-analysis method is much higher than other linear and nonlinear methods (fuzzy and neural) and has the least difference with real data. The study of the effect of oil price on Tehran Stock Exchange market stress using wavelet analysis was conducted by Jafari et al. [10]. It has been one-way relationship from the oil market to the stock market.

Neural network is one of the intelligent data mining techniques that has been used by researchers in different regions for the last 10 years. Predicting and analyzing stock market data play an important role in today's economy. The various algorithms used for prediction can be categorized into linear models (autoregressive (AR) model, moving average (MA) model, autoregressive integrated moving average (ARIMA) model) and nonlinear models (autoregressive conditional heteroskedasticity (ARCH), generalized autoregressive conditional heteroscedasticity (GARCH) model, neural network: multilayer perceptron (MLP), recursive neural networks (RNNs), long short-term memory (LSTM), and convolution neural network (CNN)) to predict a company's stock price based on historical prices. They used two different stock markets, the National Stock Exchange (NSE) of India and the New York Stock Exchange (NYSE). CNN has been found to perform better than other models. Compared with the ARIMA model, it has been observed that neural networks perform better than the existing linear model ARIMA [11, 12].

In a study conducted by Gupta and Pandey [13], the price of crude oil was predicted using frequent neural networks based on long short-term memory (LSTM). In this research, they have tried to use different types of models using different periods, revisions, and other adjustment methods, in which the result was very promising and has provided a reasonable logical forecast of crude oil prices in the near future. To increase accuracy and stability, Güleryüz and Özden [14] used LSTM and FBPr to predict future trends in Brent crude oil prices relative to previous prices and to compare two models built using data sets of 32-year weekly oil prices from June 1988 to June 2020. The model was determined to be the best fit. The data set was divided into two parts: training data and testing data, of which 25 years of 32 years have been selected as training data and the remaining 7 years as test data to confirm the accuracy of the forecast data. The coefficient of determination (R2) for LSTM and FBPr models was 0.92 and 0.89 in the training phase and 0.89 and 0.62 in the test phase, respectively. According to the results, the LSTM model has superior results for predicting oil price trends.

Salvi et al. [15] in a study examined the LSTM neural network and used it to predict the future trend of Brent oil prices based on the previous price of Brent oil. In this study, 4 types of errors have been calculated to check the accuracy of the model and errors. The mean absolute error (MAE) and root-mean-square error (RMSE) were 1.1962 and 1.9164, respectively. In a study by Chen et al. [16], using the deep learning model, they depicted the unknown complex nonlinear properties of crude oil price movement and also proposed a new model for combining crude oil price forecasting based on the deep learning model. Using the model, the major movement of crude oil prices was analyzed and modeled. The performance of the model was evaluated using price data in WTI crude oil markets. Experimental results showed that the model improves the prediction accuracy.

Moitra et al. [17] attempted to use short-term memory neural network instead of convolutional neural network to predict crude oil price. The results were promising and showed more accurate forecasts for crude oil prices in the coming days, and a hybrid model was presented for forecasting crude oil price that used sophisticated network analysis and LSTM algorithms. The research results showed that the model is more accurate and has more robustness and reliability. Aziz et al. [18] used RNN-LSTM networks to predict crude oil prices based on historical data along with other technical analysis indicators. The developed model was trained and evaluated against accuracy matrices to evaluate the network's ability to provide improved accuracy in crude oil price forecasting compared with other strategies. The result obtained from the model showed the promising ability of the RNN-LSTM algorithm to predict the movement of crude oil prices.

Jammazi and Aloui [19] predicted the global price of crude oil using empirical evidence of wavelet analysis and neural network modeling. Yao and Wang [20] proposed a multistage forecasting method based on experimental modal analysis (EMA), LSTM, and GM (1, 1) model due to the problem of crude oil price forecasting. It offered daily, weekly, and monthly crude oil prices, the results of which showed that this model has high accuracy, especially in terms of series showing long-term effects with lower frequency, and GM model (1, 1) has a good performance with the trend of forecasting crude oil prices.

Sivalingam et al. [21] used a new learning algorithm called extreme learning machine (ELM), which had good learning ability and generalizability. The period used for the study was from January 1, 2000, to April 31, 2014. Since the price of gold is related to other commodities, five commodities, including the old gold price data, the silver price, the crude oil price, the S&P 500 index, and the foreign exchange rate, were considered as inputs. This study also compared the three models such as ELM, multilayer perceptron (MLP), and radial basis function (RBF), and the results showed that the ELM algorithm has a nearly 3% increase in efficiency compared with other neural networks. Lin [22] presented how to build a gold price forecast model to understand the future trend of gold prices, using old data and the stock price technical index formula, thereby five values of the gold technical index as an independent variable and the price of gold of the next day as a dependent variable were calculated. Three prediction models including backpropagation neural network (BPN), multiple regression (MR), and principal component regression (PCR) were applied, and the results showed that the BPN model has advantage.

Mensi et al. [23] analyzed the frequency-time analysis of gold and oil prices with stock markets and a wavelet-based approach. They examined the correlations between the five major emerging stock markets: Brazil, Russia, India, China, and South Africa (BRICS) and crude oil, and Brent and gold prices. The results using the wavelet analysis approach showed that the BRICS index is correlated with the price of crude oil at low frequencies (long horizons). On the other hand, no evidence of cooperation between the BRICS stock markets and the price of gold has been found. The implications of these results for the BRICS commodity portfolio showed that portfolio risk is affected by the interaction between stocks and oil markets. Arévalo et al. [24] presented a high-frequency trading strategy using deep neural networks (DNNs). In this study, the neural network predicts the next minute. This output is converted to get the average price of the next predicted minute.

Azadeh et al. [25] designed a model for oil price forecasting. They proposed a flexible algorithm based on artificial neural network (ANN) and fuzzy regression (FR) to meet the optimal long-term oil price forecast in complex environments with uncertainty. Oil chains, crude oil distillation capacity, non-OECD oil consumption, US refinery capacity, and surplus capacity have been cited as economic indicators included in this study. Analysis of variance (ANOVA) and Duncan's multiple range test (DMRT) were then used to test the accuracy of the predictions obtained from the ANN and FR models. The result of the study was that in terms of mean percentage error (MPE), ANN models were significantly higher than FR models. Spearman's correlation test was also used.

Safari and Davallou [26] applied a hybrid model to predict oil prices. They focused on oil price forecasting due to its effect on many economic and noneconomic factors. Since factors such as economic growth, political events, and psychological expectations affect oil prices, oil price forecasting is highly uncertain. The exponential smoothing model (ESM), autoregressive integrated moving average (ARIMA), and nonlinear autoregressive (NAR) network were combined in a state-space model framework to increase prediction accuracy. Linear and nonlinear patterns have been identified in economic and financial timelines such as crude oil prices. In the proposed hybrid model (PHM), the weight of the variable time for each model was determined by the Kalman filter. PHM was used in the monthly prices of OPEC crude oil and WTI crude oil prices. Numerical results showed a reduction in prediction error using PHM compared with its constituent models, the equal weight hybrid model (EWH), the genetic algorithm weight hybrid model (GWH), and the Zhang's hybrid model (ZHM).

Ding [27] proposed a new method to predict the price of crude oil using artificial neural networks. Huang and Wang [28] presented a global crude oil price forecast and accurate estimation based on coordination using a random wavelet neural network. Yang [29] examined gold prices from July 2013 to June 2018, which aimed to analyze the daily price of gold in dollars in the first half of July 2018 with the use of the ARIMA model. In addition, the study used AC, PAC, AIC, and BIC to estimate the models, and the results suggested that ARIMA is the best model for predicting gold dollar prices.

Alameer et al. [30] proposed a new model to accurately predict monthly gold price fluctuations. In this model, a method called the whale optimization algorithm (WOA) algorithm was used as a trainer to neural network (NN) and the results were compared with other models such as NN, particle swarm optimization (PSO)-NN, genetic algorithm (GA)-NN, and grey wolf optimization (GWO)-NN. In addition, ARIMA models have been used as a criterion for evaluating the capacity of the proposed model. Experimental results showed the superiority of the WOA-NN hybrid model over other models and the proposed WOA-NN model improves the prediction accuracy obtained from the classic NN, PSO-NN, GA-NN, and GWO-NN models. ARIMA has reduced the average error. Kristjanpoller and Minutolo [31] attempted to answer the question: “Is it possible to improve the prediction of oil price fluctuations with the use of a hybrid model by combining financial variables?” The main conclusion was that the hybrid model increased the accuracy of 30% fluctuation prediction compared with previous models. The financial variables used in the model that improved the forecast were as follows: Euro/Dollar and Yen/Dollar exchange rates and DJIA and FTSE stock market indices.

Jafarzadeh Ghoushchi et al. [32] provided an extended approach to the diagnosis of tumour location in breast cancer using deep learning. This study develops a new machine learning approach based on modified deep learning (DL) to diagnose the tumour location in breast cancer. In this study, the data obtained from the databases (BCDRD01) are developed and resized and divided into data sets. A simple architecture is used for the first group of experiments, one of which utilizes a weighted function to counter the class imbalance. The results indicate that convolutional neural networks (CNNs) are an appropriate option for the separation of breast cancer lesions.

Hamdi et al. [33] investigated the relationship between oil price fluctuations and stock markets with wavelet analysis. Using quantitative regression analysis for recurring series and turbulent series during the period 2006 to 2017, the amount of fluctuations between oil prices and sectoral indicators in the Gulf Cooperation Council (GCC) countries, the United Arab Emirates, Saudi Arabia, Qatar, Oman, Kuwait and Bahrain, was examined. It was found that all sectors were dependent on oil price fluctuations. However, the banking and insurance sectors were not very sensitive to oil price fluctuations during the 10-, 25-, and 75-day periods. In addition, the relationship and the degree of interdependence between oil prices and stock returns of the sectors in the frequency domain were estimated (Table 1).

## 3. Methodology

One of the most widely used methods for modeling time series is the deep learning method. Deep learning is part of a broader family of machine learning methods based on artificial neural networks with representation learning. Deep learning architectures such as deep neural networks, deep belief networks, deep reinforcement learning, recurrent neural networks, and convolutional neural networks have been applied to fields including computer vision, speech recognition, natural language processing, machine translation, bioinformatics, drug design, medical image analysis, climate science, material inspection, and board game programs, where they have produced results comparable to and in some cases surpassing human expert performance [36]. The research process is in accordance with Table 2.

### 3.1. Collecting and Creating a Database of Oil Prices and Forming a Price Vector

The basis of modeling of forecasting system is valid, accurate, and reliable data, because erroneous data destroy all modeling validity (no matter how powerful the model is). All data used in this study are extracted from investing.com. It should be noted that this site is the first rank of Google SEO and the first rank of Alexa in investing. The data extracted for crude oil are the Brent North Sea crude oil signal.  Figure 1 shows the weekly price changes in Brent crude oil closing in the last 33 years.

As much as the data are used at a smaller sampling time (weekly, daily), high-frequency signals affect the price and the noise naturally increases and this affects the accuracy of the modeling. In other words, it has an adverse effect, but on the other hand, by increasing the number of data in smaller time intervals, more accurate information can be taught to the model.

### 3.2. Data Normalization

Normalization is the process of organizing data in a database efficiently. In other words, normalization is the way in which data are scaled. Each data set has properties that these large-value properties may have a much greater effect on the cost function than low-value properties. This problem will be solved by normalizing the properties so that their values are in the same range. The normalization operation causes all data to be in the range (1 and 0). Several statistical methods have been proposed to normalize the data. In this study, the min-max method has been used according to equation (1).  Figure 2 shows the normalized signal of Brent crude oil daily price from January 2015 to March 2021:

(1) $$\begin{array}{c} \text{x}=\frac{\text{x}-{\text{x}}_{\text{Min}}}{{\text{x}}_{\text{Max}}-{\text{x}}_{\text{Min}}}. \end{array}$$

### 3.3. Selecting the Appropriate Interval

Appropriate signal intervals should be selected for model training, validation, and testing that cover the entire signal dynamics to an acceptable level. The older the selected range, the farther it is from today's realities and naturally has adverse effects on the quality, accuracy, and precision of the model. According to the mentioned points, the selected period is a period of 6 years from January 2015 to March 2021.

### 3.4. Design and Implementation of Algorithm for Price Forecasting Process

After data collection and database creation, the amount of training and test data ratios is determined experimentally. Raw data are then standardized and thermalized. Then, the network dynamics are designed to create the necessary structure for estimating the time series. In the next step, the short-term memory network architecture is designed and the network parameters are tuned. The network quality is evaluated, and finally, the network is updated to minimize errors.

### 3.5. Modeling Using Expert Systems and Machine Learning

To predict the time series, the appropriate method for the model must be selected according to the signal behavior. There are several options for predicting a time series. Linear methods are usually the first choice in predicting time series. However, when the signal under study becomes complex and it is no longer possible to use linear methods, it is necessary to use a nonlinear method. Hence, various nonlinear methods have been developed to predict complex time series. Recursive neural tensor networks (RNTNs) including long short-term memory (LSTM) and bidirectional long-short term memory (Bi-LSTM) will be used to predict crude oil prices. The software used in this research is MATLAB R2018b.

## 4. Results

After processing the price signals and preparing them for use as a model and working on the network architecture, the proposed model with different layers and different solvents was examined. In one-layer LSTM with SGDM solver, 88% of the data is used as training data (from January 2015 to June 2020) and the remaining 12% as testing data (from June 2020 to March 2021); besides, in two-layer LSTM and three-layer LSTM with SGDM solver, 95% of the data is applied as training data (from January 2015 to January 2021) and the remaining 5% as testing data (from January 2021 to March 2021), which are shown in Figures 3–5.

In one-layer LSTM with RMSProp solver, 90% of the data is used as training data (from January 2015 to July 2020) and the remaining 10% as testing data (from July 2020 to March 2021), which is shown in Figure 6.

In one-layer LSTM with the Adam solver, 90% of the data is used as training data (from January 2015 to July 2020) and the remaining 10% as testing data (from July 2020 to March 2021), which is shown in Figure 7.

Initially, with only one-layer LSTM with SGDM solver, the root-mean-square error (RMSE) is equal to 1.88, maximum error is equal to 5.82, modeling time is equal to 429 seconds, mean squared error (MSE) is equal to 3.9, the number of feedback regressors is [1, 2, 3, 4], and the number of hidden layers is 100, which are shown in Table 3. Figures 8 and 9, respectively, provide comparison of system response to real observations and comparison of system response to real observations (up-close) and their error.

Then, to improve the model error, the one-layer LSTM was changed to Bi-LSTM with SGDM solver. It is indicated that the RMSE is equal to 2.1838, maximum error is equal to 7.74, modeling time is equal to 822 seconds, MSE is equal to 3.60, the number of feedback regressors is [1, 2, 3, 4], and the number of hidden layers is 100, which are shown in Table 4. Figures 10 and 11, respectively, provide comparison of system response to real observations and comparison of system response to real observations (up-close) and their error.

By Bi-LSTM with SGDM solver, it is indicated that the RMSE is equal to 1.94, maximum error is equal to 11.24, modeling time is equal to 114 seconds, MSE is equal to 3.72, the number of feedback regressors is [1, 2], and the number of hidden layers is 10, which are shown in Table 5. Figures 12 and 13, respectively, provide comparison of system response to real observations and comparison of system response to real observations (up-close) and their error.

A Bi-LSTM layer with the Adam solver, like the previous case, did not have acceptable results for model evaluation and is not a suitable solvent.

Then, to improve the results, another LSTM layer was added to the previous layer, so that the model error might be corrected. It is shown that the RMSE is equal to 1.53, maximum error is equal to 7, modeling time is equal to 345.32 seconds, MSE is equal to 2.68, the number of feedback regressors is [1, 2], and the number of hidden layers is 80, which are shown in Table 6. Figures 14 and 15, respectively, provide comparison of system response to real observations and comparison of system response to real observations (up close) and their error.

Finally, the model with three-layer LSTM was tested with SGDM solver, whose RMSE is equal to 1.58, maximum error is equal to 5, modeling time is equal to 911 seconds, MSE is equal to 2.70, the number of feedback regressors is [1, 2, 3], and the number of hidden layers is 80, which are shown in Table 7. Figures 16 and 17, respectively, provide comparison of system response to real observations and comparison of system response to real observations (up-close) and their error.

At the end and in Table 8, all the models are compared with each other and they can be checked with the parameters. Two-layer LSTM with SGDM solver has less RMSE and MSE, and as a result the accuracy of the model is higher and better, but in terms of modeling time, one-layer LSTM with RMSProp solver is a more suitable option. To compare the number of hidden layers, one-layer LSTM with RMSProp solvent and a bi-LSTM layer with RMSProp solvent have fewer hidden layers, which again makes one-layer LSTM a better option than the Bi-LSTM layer.

## 5. Conclusion

The main question of this research was as follows: “How can the price of time secret data be predicted by the deep learning method?” The answer was presented by collecting an appropriate database, reviewing and selecting modeling methods and efficient algorithms appropriate to the type of signal, and identifying as many effective factors and parameters as possible. It is indicated that the price of Brent crude oil in the global market can be predicted.

Then, in response to the question “How much does the future price of Brent crude oil depend on its past price?” different answers were given in different models, but by comparing the models, it is concluded that the price of crude oil is dependent on the price of at least two days ago. The question then arose, “Does the future price of Brent crude oil depend on external factors related to it?” Examining the external signals, it was found that the price of crude oil is correlated with the factors and prices of other signals, such as gold and the Canadian dollar. Finally, in response to the question “Does the performance of an expert system depend on the quality of its training?” comparing the models, especially the neural network models with the recurrent and feed-forward training structures, it can be concluded that the performance of expert systems in the field of machine learning is highly dependent on the type and quality of their training.

In this study, first by collecting daily data from a reliable source, a database was formed to model and predict the price of Brent crude oil signals. The data period for modeling was selected from January 2015 to March 2021.

In this study, deep learning method was used to model and predict the price of Brent crude oil price signals. The reason for choosing this method was the complex dynamics of price signals and the lack of accurate information. Nonlinear techniques of artificial neural networks and deep learning were used for modeling. Then, the network architecture was worked on and the model error rate was evaluated by comparing different layers and solvents such as SGDM, RMSProp, and Adam. The superiority of SGDM solvent over others was shown, and finally, it can be mentioned as the superior method of modeling of price forecasting in Brent crude oil field.

The following points are summarized from this research:

- Crude oil price signals exhibit highly nonlinear and complex behavior
- The SGDM solvent has less error in predicting Brent crude oil price for the designed model than RMSProp and Adam solvent
- The RMSProp solvent also has less error than the Adam solvent in predicting Brent crude oil price for the designed model
- By adding an LSTM layer to the network structure, the error model was improved, resulting in a more accurate result
- LSTM layers perform better than Bi-LSTM layers and further reduce model error

### 5.1. Contributions

- In this study, unlike all previous studies on Brent crude oil forecasting, the model network architecture has been worked on and an attempt has been made to improve the model error by changing layers and solvents. Other research differs from that conducted in this study. For example, in a study by Chen et al. [16], using a deep learning model, complex nonlinear features of unknown crude oil price movements were depicted. Also, a new model is proposed for crude oil price forecasting based on the deep learning model, which differs from the method used in this study.
- Moitra et al. [17], in a study entitled “Crude oil price prediction using the LSTM method,” have tried to use short-term memory neural network instead of convolutional neural network to predict crude oil price. They have used complex network analysis and LSTM and deep learning algorithms, while in this study we authors tried to provide a better and more appropriate model by changing the LSTM layer to the Bi-LSTM layer.
- Furthermore, in existing studies no comparison was made to present and select the best model in the field of Brent crude oil price forecasting.

Brokers, traders, and investment advisers working in the field of energy, especially oil, are advised to predict the price of oil and take risk hedging measures to actively manage their portfolio using this model.

To improve the quality of this research, suggestions for future studies are presented, which are as follows:

- Designing a crude oil price forecasting model with other neural networks
- Using other data processing methods such as STFT on crude oil signal and comparing results

Constraints are an integral part of research. However, in general, the limitations of research included the following:

- The strong dependence of the results on the type of modeling
- Coronavirus pandemic during the research period

## Figures and Tables

**Figure 1:** Weekly price changes in Brent crude oil closing in the last 33 years.

**Figure 2:** Normalized signal of Brent crude oil daily price from January 2015 to March 2021.

**Figure 3:** Training and test data for one-layer LSTM modeling with SGDM solver.

**Figure 4:** Training and test data for two-layer LSTM modeling with SGDM solver.

**Figure 5:** Training and test data for three-layer LSTM modeling with SGDM solver.

**Figure 6:** Training and test data for one-layer LSTM modeling with RMSProp solver.

**Figure 7:** Training and test data for one-layer LSTM modeling with the Adam solver.

**Figure 8:** Comparison of system response to real observations of one-layer LSTM with SGDM solver.

**Figure 9:** Comparison of system response to real observations (up-close) of one-layer LSTM with SGDM solver and their error.

**Figure 10:** Comparison of system response to real observations of Bi-LSTM with SGDM solver.

**Figure 11:** Comparison of system response to real observations (up-close) of Bi-LSTM with SGDM solver and their error.

**Figure 12:** Comparison of system response to real observations of Bi-LSTM with RMSProp solver.

**Figure 13:** Comparison of system response to real observations (up-close) of Bi-LSTM with RMSProp solver and their error.

**Figure 14:** Comparison of system response to real observations of two-layer LSTM with SGDM solver.

**Figure 15:** Comparison of system response to real observations (up-close) of two-layer LSTM with SGDM solver and their error.

**Figure 16:** Comparison of system response to real observations of three-layer LSTM with SGDM solver.

**Figure 17:** Comparison of system response to real observations (up-close) of three-layer LSTM with SGDM solver and their error.

**Table 1:** Comparison of research tools conducted in previous years in the field of price forecasting.

No.		Nonlinear time series	Linear time series	IO-nonlinear model	IO-linear model	Deep learning	MLP NN	Oil	Gold
1	Azadeh et al. [25]			*∗*		*∗*		*∗*	
2	Li [34]			*∗*			*∗*		*∗*
3	Kristjanpoller and Minutolo [31]			*∗*			*∗*		*∗*
4	Lin [22]			*∗*	*∗*		*∗*		*∗*
5	Mensi et al. [23]	*∗*	*∗*					*∗*	*∗*
6	Arévalo et al. [24]						*∗*	*∗*	
7	Safari and Davallou [26]	*∗*	*∗*			*∗*		*∗*	
8	Chen et al. [16]					*∗*			
9	Gupta and Pandey [13]					*∗*			
10	Yang [29]		*∗*						*∗*
11	Ding [27]			*∗*			*∗*	*∗*	
12	Huang and Wang [28]			*∗*			*∗*	*∗*	
13	Hiransha et al. [11]					*∗*			
14	Alameer et al. [30]	*∗*	*∗*				*∗*		*∗*
15	Salvi et al. [15]					*∗*			
16	Güleryüz and Özden [14]					*∗*			
17	Wu et al. [35]					*∗*			
18	Moitra et al. [17]					*∗*			

**Table 2:** Research process.

No.	Activity
1	Collecting and creating an oil price database and forming a price vector
2	Normalization of raw data
3	Preprocessing
4	Selecting the appropriate interval
5	Design and implementation of algorithms for price prediction process
6	Modeling using expert systems and machine learning
7	Identifying external signals affecting crude oil price output
8	Comparison of models

**Table 3:** Results of one-layer LSTM with SGDM solver for Brent crude oil.

Parameter	Value
Root-mean-square error (RMSE)	1.88
Maximum error	5.825
Modeling time	429
Mean squared error (MSE)	3.9
Feedback regressors	[1 2 3 4 ]
Hidden layers	100

**Table 4:** Results of Bi-LSTM with SGDM solver.

Parameter	Value
Root-mean-square error (RMSE)	2.18
Maximum error	7.74
Modeling time	822
Mean squared error (MSE)	3.60
Feedback regressors	[1 2 3 4 ]
Hidden layers	100

**Table 5:** Results of Bi-LSTM with RMSProp solver.

Parameter	Value
Root-mean-square error (RMSE)	1.94
Maximum error	11.24
Modeling time	114
Mean squared error (MSE)	3.72
Feedback regressors	[1, 2]
Hidden layers	10

**Table 6:** Results of two-layer LSTM with SGDM solver.

Parameter	Value
Root-mean-square error (RMSE)	1.53
Maximum error	7
Modeling time	345.32
Mean squared error (MSE)	2.68
Feedback regressors	[1, 2]
Hidden layers	80

**Table 7:** Results of three-layer LSTM with SGDM solver.

Parameter	Value
Root-mean-square error (RMSE)	1.58
Maximum error	5
Modeling time	911
Mean squared error (MSE)	2.70
Feedback regressors	[1, 2, 3]
Hidden layers	80

**Table 8:** Comparison of modeling results.

Parameter	One-layer LSTM with SGDM solver	One-layer LSTM with RMSProp solver	One-layer LSTM with Adam solver	A Bi-LSTM with SGDM solver	A Bi-LSTM with RMSProp solver	Two-layer LSTM with SGDM solver	Three-layer LSTM with SGDM solver
RMSE	1.88	1.59	2.73	2.18	1.94	1.53	1.58
Maximum error	5.825	12.44	17.31	7.74	11.24	7	5
Modeling time	429	63.75	248	822	114	345.32	911
MSE	3.9	3.36	5.76	3.60	3.72	2.68	2.70
Feedback regressors	[1, 2, 3, 4]	[1, 2, 3, 4]	[1, 2, 7]	[1, 2, 3, 4]	[1, 2]	[1, 2]	[1, 2, 3]
Hidden layers	100	10	80	100	10	80	80

## Data Availability

The data that support the findings of this study are available from the corresponding author upon reasonable request.
